The article "LncRNA PFAR contributes to fibrogenesis in lung fibroblasts through competitively binding to miR-15a" was published in 2019. Journal: Biosci Rep.

# LncRNA PFAR contributes to fibrogenesis in lung fibroblasts through competitively binding to miR-15a

**DOI:** 10.1042/BSR20190280

**Published:** 2019-07-19

**Authors:** Jian Sun, Wei Su, Xiaoguang Zhao, Tianjiao Shan, Tongzhu Jin, Yingying Guo, Chao Li, Ruotong Li, Yuhong Zhou, Hongli Shan, Xiaohan Sun, Haihai Liang

**Affiliations:** 1 Department of Pharmacology (State-Province Key Laboratories of Biomedicine-Pharmaceutics of China, Key Laboratory of Cardiovascular Research, Ministry of Education), College of Pharmacy, Harbin Medical University, Harbin, Heilongjiang 150081, P. R. China; 2 Northern Translational Medicine Research and Cooperation Center, Heilongjiang Academy of Medical Sciences, Harbin Medical University, Harbin, Heilongjiang 150081, P. R. China; 3 Department of Pediatrics, The Second Affiliated Hospital of Harbin Medical University, Harbin, Heilongjiang 150086, P. R. China

**Keywords:** fibroblasts, large intervening non-coding RNA, microRNA

## Abstract

Idiopathic pulmonary fibrosis (IPF) is a chronic, progressive, debilitating disease with unknown etiopathogenesis. Previous reports have reported that long non-coding RNAs (lncRNAs) were involved in various pathophysiological processes. However, the role of lncRNAs in IPF has not been fully described. We aimed to explore the relationship between miR-15a and lncRNA PFAR and its function in pulmonary fibrosis. Biological information analysis and luciferase were used to identify targeted binding of lncRNA PFAR and miR-15a. Western blot, quantitative reverse transcription-PCR (qRT-PCR) and immunofluorescence staining were conducted to detect fibrosis-related factors. Fibroblasts proliferation were analyzed using 5-ethynyl-2′-deoxyuridine (EdU) staining and fibroblasts migration ability were measured using wound-healing scratch assay. We identified that lncRNA PFAR has a binding site with miR-15a and luciferase reporter assays demonstrated their combinative relationship. Our results showed that silencing PFAR attenuated TGF-β1 induced fibrogenesis in primary lung fibroblasts. And miR-15a antagonized the function of PFAR and inhibited PFAR induced extracellular collagen deposition, fibroblasts proliferation, migration and differentiation. In conclusion, our results revealed that PFAR functions as a competitive endogenous RNA (ceRNA) by acting as a sponge for miR-15a, revealing a potential regulatory network involving PFAR and miR-15a with a role in the modulation of YAP1-Twist expression. This mechanism may contribute to a better understanding of pulmonary fibrosis pathogenesis and treatment method.

## Introduction

Idiopathic pulmonary fibrosis (IPF), the most common idiopathic interstitial pneumonia, is characterized by cell proliferation, interstitial inflammation, fibrosis, or a combination of these symptoms not caused by infection or cancer [1]. Due to the high mortality rate of pulmonary fibrosis, new treatments and biomarkers are needed to be elucidated [2,3]. In the past few decades, research has explored the mechanisms of IPF and showed that the pathogenesis and progression of IPF are closely related to persistent epithelial damage and dysfunction between epithelial and mesenchymal cells after fibroblast activation [4–6]. Both Pirfenidone and Nintedanib are oral anti-fibrotic drugs that have been shown to slow disease progression and improve progression-free survival, presenting new hopes for patients with IPF, but also with limitations [7,8]. Therefore, it is crucial to deeply explore the pathogenesis of IPF and provide a theoretical basis for disease treatment. In recent years, the non-coding human transcriptome has emerged as a new opportunity for the development of novel therapeutic strategies and biomarker discovery.

MicroRNAs are being considered as a novel type of bio-markers and potential therapeutic targets for various diseases [9]. There is now increasing evidence indicate that the expression of miRNAs is altered in the airways and lungs of patients with a broad range of respiratory diseases [10]. Our previous study has found that miR-15a inhibits lung fibroblast activation and fibrogenesis by regulating the YAP1-Twist axis. However, the upstream factors that regulating dysregulation of miR-15a in lung fibrosis remains to be elucidated. LncRNAs (long non-coding RNAs), defined as non-coding RNA transcripts longer than 200 nt, are emerging key regulators of diverse cellular processes through acting as endogenous decoys that compete with miRNA [11]. The dysfunction of lncRNAs is closely related to various hereditary diseases, autoimmune diseases, metabolic diseases and tumors. In addition, lncRNAs were also recently recognized as functional regulators of fibrosis [12].

In the present study, we investigated the roles of lncRNA PFAR and miR-15a in TGF-β1 induced lung fibrogenesis and found that miR-15a is necessary for the pro-fibrotic effects of PFAR in lung fibrosis.

## Materials and methods

### Animal model and treatment

Adult male C57BL/6 mice at 6–8 weeks of age were purchased form Vital River Laboratory Animal Technology (Beijing, China), and all the experiments were performed in accordance with the Ethics Committees of Harbin Medical University. The mice were anesthetized with amobarbital (40 mg/kg, intravenously [i.v.]). The interfered sequence of lncRNA-PFAR packaged in the adenovirus-associated virus 5 (AAV5) was intratracheally injected to mice.

### Cell culture

Primary lung fibroblasts were isolated from lungs of 1–3 days old, Kunming mice. In brief, lungs were placed on Petri dishes with DMEM (Biological Industries, Israel) and continuously minced with a sterile razor blade until a homogenous mixture was achieved. The minced lung tissue was digested with trypsin (0.5 mg/ml). The cells were precipitated by centrifugation and cultured with complete medium (89% DMEM + 10% FBS + 1% Penicillin–Streptomycin solution). After 6 h, the non-adherent cells were removed. Cells were placed in a standard humidity incubator with a temperature of 37°C and containing 5% of CO_2_. The final concentration of TGF-β1 (Sigma–Aldrich, U.S.A.) was 10 ng/ml. The cells were cultured in the medium containing TGF-β1 for 48 h before being collected for further analysis.

### Western blot

Cells were lysed with RIPA lysis buffer (Beyotime, Jiangsu, China). A total of 40 μg of protein was run on a 10% SDS-polyacrylamide gel. After being electrophoretically transferred to a pure nitrocellulose blotting membrane (Pall Life Sciences, Ann Arbor, MI, U.S.A.), the proteins were probed with primary antibodies, with β-actin as an internal control. Primary antibody against Twist were purchased from Wanlei biotechnology (Liaoning, China). Primary antibody against α-smooth muscle actin (SMA) was purchased from Abcam (Abcam Inc., U.S.A.). Primary antibodies against YAP1, collagen 1 or fibronectin 1 (FN1) were purchased from Proteintech (Wuhan, China). The immunoreactivity was detected using Odyssey Infrared Imaging System (Odyssey CLx, Biosciences, U.S.A.). The Western blot bands were quantified using Image Studio Ver 5.2 software and normalized with respect to loading control.

### Quantitative reverse transcription-PCR

Total RNA from collected cells or tissues were extracted using TRIzol reagent. The growth media were removed from the culture dish. Approximately 1 ml of TRIzol was directly added to each well, and the cell lysis was achieved by repeatedly grinding. The cells were incubated at room temperature for 5 min. Afterward, 250 μl of chloroform was added to each sample. The samples were incubated for 10 min at room temperature and subsequently centrifuged at 13,500 ***g*** at 4°C for 15 min. The samples were divided into three layers. The aqueous phase was mixed with 500 μl of isopropyl alcohol at room temperature for 35 min. The samples were centrifuged at 13,500 ***g*** at 4°C for 10 min, and removed the supernatant. The RNA pellet was gently washed with 1 ml of ethanol, centrifuged at 10,600 ***g*** for 5 min at 4°C, and resuspended in 10 μl of RNA-free water. NanoDrop 8000 (Thermo, U.S.A.) was used to determine the concentration and purity of the extracted RNAs. The relative expression levels of mRNAs and miRNAs were quantified by the mirVana™ quantitative reverse transcription-PCR (qRT-PCR) miRNA Detection Kit and quantitative RT-PCR with SYBR Green I (Applied Biosystems, Foster City, CA). The relative expression levels were calculated based on *C*_t_ values and were normalized to the U6 or GAPDH levels of each sample, respectively.

### miRNA and plasmid transfection

The primary lung fibroblasts were plated in six-well dishes (2 × 10^5^ cells per well) until the cell density reached 70–80% prior to small RNA transfection. On the following day, cells were washed with serum-free medium once and then incubated with serum-free medium for 6 h. The miRNAs/plasmid and Lipofectamine 2000 (Invitrogen, Carlsbad, CA) were separately mixed with Opti-MEM^®^ I Reduced Serum Medium (Gibco, Grand Island, NY) for 5 min. Then, the two mixtures were combined and incubated at room temperature for 20 min. The Lipofectamine miRNAs/plasmid mixture was added to the cells and incubated at 37°C for 6 h. Subsequently, 2 ml fresh medium containing 10% FBS was added to the each well and the cells were maintained in the culture until following experiments.

### Immunofluorescence staining

Approximately 2 × 10^5^ primary lung fibroblasts cells were cultivated in a 24-well plate. After transfection and TGF-β1 treatment, these cells were rinsed with cold phosphate-buffered saline (PBS) for three times and fixed in 4% paraformaldehyde for 30 min. The cells were rinsed with PBS for three times, incubated with 0.4% Triton X-100 for 1 h at room temperature, and blocked with 50% normal goat serum for 1 h at 37°C. Afterward, α-SMA antibody (1:200, Abcam, U.S.A.) or Vimentin antibody (1:200, Proteintech, Wuhan,China) was added dropwise into each well at 4°C overnight. Subsequently, incubated with FITC-conjugated goat anti-mouse or goat anti-rabbit antibody for 1 h. All operating steps were conducted in the dark because fluorescent secondary antibodies were added. After rinsing with PBS for three times, the nuclei were stained with DAPI (Roche Molecular Biochemicals, Basel, Swizerland) for 5 min at room temperature. Immunofluorescence was analyzed under a fluorescence microscope (Olympus, IX73, Japan).

### 5-ethynyl-2′-deoxyuridine assay

The cell proliferation was tested by EdU (5-ethynyl-20-deoxyuridine) assay using Cell-Light EdU DNA Cell Proliferation Kit (RiboBio, Guangzhou, China). Primary lung fibroblasts (1 × 10^5^) were seeded in each well of 24-well plates for transfection with PFAR/sh-PFAR, miR-15a mimics/inhibitor or negative control (NC) oligonucleotide. After incubation at 37°C and 5% CO_2_ for 48 h, cells were added with 200 μl 50 μM EdU and incubated for another 2 h. Cells were then fixed with 4% paraformaldehyde and stained with Apollo Dye Solution for proliferating cells. Nucleus in all cells were stained with DAPI. The cell proliferation rate was calculated according to the manufacturer’s instructions. Images were taken using a fluorescence microscope (Olympus, IX73, Japan).

### Wound-healing scratch assay

To evaluate the cell migration consistent with the wound healing properties of fibroblasts, an *in vitro* scratch assay was performed, the primary lung fibroblasts were seeded with 50,000 cells/cm^2^ in six-well plates. When the cells formed a confluent monolayer, they were scratched with a 2-μl pipette tip, and washed in PBS to remove cell debris. The scratch was visualized using phase-contrast microscopy (×20 objective) and photographed, and the width of the wound was measured at 0h, 24h and 48 h. A line was drawn along each side of the scratch to remove minor irregularities generated by the mechanical scratch from the pipette tip, and the distance between the lines measured at 4 separate points. The relative wound size at each time point was analyzed by ImageJ (http://imagej.nih.gov/ij/). Each variant of stimulation was done in four technical replicates.

### Luciferase reporter assays

Sequences of the lncRNA PFAR containing wild-type (WT) or mutated miR-15a binding sites were synthesized by Invitrogen and amplified by PCR. The PCR fragments were subcloned into the SacI and HindIII sites downstream of the luciferase gene in the pMIR-Report plasmid (Promega). A miR-15a sensor reporter was constructed according to the method described previously [13]. HEK293T cells or lung fibroblasts were co-transfected with 0.1 μg of the luciferase-PFAR chimeric vector and miR-15a mimic by lipofectamine 2000 (Invitrogen, U.S.A.). We collected the cell lysis after 24-h transfection and measured luciferase activities with a dual luciferase reporter assay kit (Promega, U.S.A.).

### Statistical analysis

Data were presented as mean ± SEM of at least three independent experiments. Unpaired Student’s *t*-test was used to compare the two groups. *P*<0.05 was considered to indicate statistical significance.

## Results

### LncRNA PFAR binds to miR-15a and regulates its activity

To delineate the molecules that regulate miR-15a in lung fibrosis, we first used the bioinformatics analysis to predict upstream factor of miR-15a and found that miR-15a has a binding site with lncRNA PFAR. Then, we knocked down PFAR in mice by intratracheal injection of AAV5 containing a short hairpinRNA (shRNA) against PFAR (AAV5-sh-PFAR) to evaluate whether PFAR regulates the expression of miR-15a. As shown in Figure 1A, injection of AAV5-sh-PFAR promoted the expression of miR-15a in the lungs of mice. Next, we transfected PFAR-overexpression or sh-RNA plasmid into lung fibroblasts to examine the effect of PFAR on miR-15a. We found that silencing PFAR promoted the expression of miR-15a, whereas overexpression of PFAR resulting to decreased expression of miR-15a (Figure 1B,C).

**Figure 1:** LncRNA PFAR acts as molecular sponge of miR-15a (**A**) qRT-PCR analysis of the expression of miR-15a in the lungs of mice after injection of AAV5-sh-PFAR. qRT-PCR analysis of the expression of miR-15a in lung fibroblasts after PFAR inhibition (**B**) or overexpression (**C**). (**D**) Predicted binding sites of PFAR and miR-15a. PFAR-Mut, mutated binding site. (**E**) Luciferase reporter activities of chimeric vectors carrying the luciferase gene and a fragment of PFAR containing WT or mutated miR-15a-binding site. (**F**) Lung fibroblasts were co-transfected with the miR-15a sensor and PFAR/sh-PFAR and its corresponding scrambled form, and luciferase activity was detected. (**G**) Lung fibroblasts were co-transfected with the miR-15a sensor, miR-15a and PFAR and its corresponding scrambled form, and luciferase activity was detected. All data are presented as mean ± SEM. *n*=6 independent experiments. ^*^P<0.05; NS, not significant.

To better understand the relation between PFAR and miR-15a, we constructed a miR-15a sensor luciferase vector containing a perfect miR-15a target site that was incorporated into the 3′UTR of the luciferase gene, a strategy that has been widely used in our previous study [13]. Further evidence was generated from our experiments with the luciferase vector carrying a PFAR fragment encompassing WT or mutated binding sites for miR-15a (Figure 1D). As illustrated in Figure 1E, miR-15a suppressed the luciferase activity with WT PFAR (PFAR-WT) but not with mutated PFAR vector in HEK293T cells. However, miR-15a lost its inhibitory effect with mutated PFAR (mutation of binding sites for miR-15a). As shown in Figure 1F, the luciferase activity of the miR-15a sensor was increased in lung fibroblasts transfected with PFAR, indicating that PFAR bound miR-15a to limit the inhibitory effect of the latter on luciferase activity. In contrast, silencing of PFAR by shRNA inhibited the luciferase activity of the miR-15a sensor. Moreover, overexpression of PFAR alleviated the inhibitory effect of miR-15a on its sensor (Figure 1G).

### MiR-15a is involved in PFAR-induced collagen deposition

Interstitial pneumonia is characterized by pathological proliferation of mesenchymal cells and uncoordinated collagen deposition [14]. We found that overexpression of PFAR increased collagen 1α1 and collagen 3α1 at mRNA levels, whereas these effects were abrogated by enhanced expression of miR-15a (Figure 2A,B). Meanwhile, miR-15a also inhibited collagen 1α1 protein levels induced by PFAR detecting with Western blot (Figure 2C). In addition, we used shRNA to inhibit PFAR expression in lung fibroblasts. The data from Figure 2D–F showed that knockdown of PFAR inhibited TGF-β1-induced collagen production in both mRNA and protein levels in lung fibroblasts, whereas this effect was alleviated by the inhibition of miR-15a.

**Figure 2:** miR-15a is necessary for the PFAR-induced collagen deposition (**A,B**) qRT-PCR was used to determine the effect of PFAR overexpression on collagen 1α1 and collagen 3α1 production in lung fibroblasts. (**C**) Western blot analysis of collagen1α1 in lung fibroblasts after transfection of PFAR. The mRNA levels of collagen 1α1 (**D**) and collagen 3α1 (**E**) were measured by qRT-PCR in PFAR-depleted lung fibroblasts treated with TGF-β1. (**F**) Western blot analysis of collagen 1α1 in TGF-β1-treated lung fibroblasts after PFAR silencing. All data are presented as mean ± SEM. *n*=4 independent experiments. ^*^P<0.05.

### MiR-15a mediates the proliferative effect of PFAR in lung fibroblast

It has been reported that the number of subepithelial fibroblast foci, which are clusters of fibroblasts in the extracellular matrix (ECM), correlate with IPF prognosis and survival [15]. We further explored whether PFAR regulates fibroblasts proliferation via miR-15a *in vitro*. We conducted the EdU staining and scratch wound-healing assay to detect the ability of cell proliferation and migration. As illustrated in Figure 3A,B, forced expression of PFAR promoted cell proliferation and migration whereas these effects were nearly ameliorated by overexpression of miR-15a. Conversely, we also found that inhibition of PFAR mitigated the TGF-β1-induced proliferation and migration, whereas these effects were effectively reversed with the simultaneous expression of the miR-15a inhibitor (Figure 3C,D).

**Figure 3:** PFAR acts as a regulator for miR-15a to promote lung fibroblasts proliferation (**A**) EdU staining demonstrated the effect of PFAR on lung fibroblast proliferation. Scale bar, 50 μm. (**B**) Scratch assay for the evaluation of migration of lung fibroblasts after PFAR overexpression. Scale bar, 200 μm. (**C**) EdU staining demonstrates the effect of PFAR inhibition on lung fibroblast proliferation. Scale bar, 50 μm. (**D**) Scratch assay for the evaluation of migration of lung fibroblasts after PFAR depletion. Scale bar, 200 μm. All data are presented as mean ± SEM. *n*=4 independent experiments. ^*^P<0.05.

### PFAR regulates the TGF-β1-induced fibroblast differentiation through the miR-15a

Fibroblast-to-myofibroblast trans-differentiation is a process involved in the pathogenesis of lung fibrosis [16]. We then used immunofluorescence experiments to detect α-SMA-positive myofibroblast formation to evaluate the ability of cell differentiation. As shown in Figure 4A,B, forced expression of PFAR promoted fibroblast–myofibroblast transition; however, it was significantly alleviated after overexpression of miR-15a. On the contrary, silencing PFAR inhibits TGF-β1-induced fibroblast–myofibroblast differentiation, and this effect was reversed by miR-15a inhibitor (Figure 4C,D).

**Figure 4:** PFAR promotes fibroblast–myofibroblast transition by modulating the function of miR-15a (**A**) Effect of PFAR on lung fibroblast–myofibroblast transition, as measured by immunofluorescence. Scale bar, 50 μm. (**B**) Western blot analysis of α-SMA in lung fibroblasts after transfection of PFAR. (**C**) Effect of PFAR knockdown on myofibroblast formation, as measured by immunofluorescence. Scale bar, 50 μm. (**D**) Western blot analysis of α-SMA proteins in TGF-β1-treated lung fibroblasts after PFAR silencing. (**E**) Western blot analysis of YAP1 and Twist proteins in lung fibroblasts after transfection of PFAR. (**F**) Western blot analysis of YAP1 and Twist proteins in TGF-β1-induced lung fibrogenesis after PFAR silencing. All data are presented as mean ± SEM. *n*=4 independent experiments. ^*^P<0.05.

In our previous study, we found that miR-15a participates in the pulmonary fibrosis process by regulating YAP1-Twist axis. As shown in Figure 4E,F, Overexpression of miR-15a inhibited PFAR-induced up-regulation of YAP1 and Twist at protein levels. Consistent with the above, inhibition of PFAR mitigated the TGF-β1-induced YAP1 and Twist protein levels, but reversal after giving miR-15a inhibitor.

## Discussion

In the present study, we found that lncRNA PFAR participates in pulmonary fibrosis by binding to miR-15a and regulating the expression of its downstream target YAP1 (Figure 5). These results uncover a regulatory network in pulmonary fibrosis and shed light on the function of lncRNAs and their relationship with miRNAs and their targets.

**Figure 5:** Proposed model for the mechanism involving PFAR and miR-15a in lung fibrosis lncRNA PFAR promoted lung fibroblasts activation and ECM deposition via regulating of YAP1-Twist axis by acting as a sponge of miR-15a, whereas knockdown of PFAR exerted the anti-fibrotic effect.

The lungs are constantly exposed to many injuries but repetitive alveolar epithelial injury could result in epithelial cell senescence and pro­fibrotic epigenetic reprogramming, leading to a maladaptive response of IPF [17]. Epithelial activation is followed by a dynamic and complex process characterized by the migration and proliferation of fibroblasts and their differentiation to myofibroblasts, a critical process for the development of fibrosis through excessive ECM deposition [18]. These possible pathological mechanisms are potential ways for treatment of IPF.

It is well accepted that miRNAs are key factor in the pathogenesis of IPF in both human and experimental animal lung diseases. Recent studies demonstrating that miRNAs were involved in the initiation and progression of IPF and used as targets for the treatment of lung fibrosis [19]. MiR-26a had been identified as an anti-fibrotic effector in IPF targeting regulation of CTGF, HMGA2 and Lin28B in our previous studies [20–22]. MiR-15a targets YAP1 to inhibit pulmonary fibrosis both *in vivo* and *in vitro* experiments. As an endogenous competitive RNA, lncRNA is gradually discovered in fibrosis. Recent studies from our group have found that inhibition of lncRNA PFRL prevents pulmonary fibrosis by disrupting the miR-26a/Smad2 loop [23], and lncRNA PFAL promotes lung fibrosis through CTGF by competitively binding miR-18a [24]. Liu et al. [25] reported that silencing lncRNA PCF by directly targeting miR-344a-5p alleviates pulmonary fibrosis in rats. Liu et al. [26] found that LncRNA-ATB promotes EMT during silica-induced pulmonary fibrosis by competitively binding miR-200c. A recent study shows that kidney-enriched lnc-TSI inhibits renal fibrogenesis by negatively regulating the TGF-β/Smad3 pathway, a classic pathway involved in the development of pulmonary fibrosis [27], indicating the important role of lncRNA in fibrotic lesions.

We have verified the role of PFAR in promoting cell proliferation and ECM deposition in pulmonary fibrosis, and considered PFAR as a new strategy for prevention and treatment of pulmonary fibrosis [13]. Our results demonstrated that lncRNA PFAR contains the binding sites for several key miRNAs such as miR-138 and miR-15a. We speculate that PFAR may provide a more effective strategy for the treatment of lung fibrosis.

The limitations to the present study are also worth of attention. We only verified the effects of lncRNA PFAR and miR-15a on primary lung fibroblasts, rather than detect other cell types in the lungs. Knocking down PFAR in mice may cause different reactions in epithelial cells, which requires further research and verification. Further studies are needed to verify whether PFAR can be a therapeutic target in human IPF.

## Conclusions

Our study identified that lncRNA PFAR acts as an endogenous sponge of miR-15a and regulate fibrogenesis in lung fibroblasts. These findings provide novel information for understanding the mechanisms underlying PFAR-mediated tissue fibrosis. Our work hints the possibility of a new therapeutic target to halt the damaging process in diseases, although this remains to be confirmed by future studies.

## Abbreviations

AAV5: adenovirus-associated virus 5
ECM: extracellular matrix
EdU: 5-ethynyl-2′-deoxyuridine
IPF: idiopathic pulmonary fibrosis
i.v.: intravenously
LncRNA: long non-coding RNA
PBS: phosphate-buffered saline
qRT-PCR: quantitative reverse transcription-PCR
shRNA: short hairpinRNA
SMA: smooth muscle actin
WT: wild-type
